The article "Artificial Intelligence-Based CT Imaging on Diagnosis of Patients with Lumbar Disc Herniation by Scalpel Treatment" was published in 2022. Journal: Comput Intell Neurosci.

# Artificial Intelligence-Based CT Imaging on Diagnosis of Patients with Lumbar Disc Herniation by Scalpel Treatment

**DOI:** 10.1155/2022/3688630

**Published:** 2022-05-27

**Authors:** Xiaofei Fan, Xiaoming Qiao, Zhisheng Wang, Luetao Jiang, Yue Liu, Qingshan Sun

**Affiliations:** ^1^Department of Medicine, Shandong Medical College, Jinan 250002, Shandong, China; ^2^Department of Orthopedics, The Affiliated Suqian Frist People's Hospital of Nanjing Medical University, Suqian 223899, Jiangsu, China; ^3^Department of Endocrinology and Metabolism, Affiliated Hospital of Guizhou Medical University, Guiyang 550001, Guizhou, China; ^4^Department of Medical Administration, Shandong Provincial Third Hospital, Jinan 250031, Shandong, China

## Abstract

The aim of this study was to explore the application effect of computed tomography (CT) image based on active contour segmentation algorithm in the treatment of lumbar disc herniation (LDH) with scalpel. 78 patients with LDH were selected and divided into a lateral crypt block treatment group (group A) and a scalpel treatment group (group B) randomly. All the patients were examined by lumbar CT images based on artificial intelligence (AI) algorithm. Then, the clinical efficacy and Japanese orthopedic association (JOA) and visual analogue scale (VAS) scores were compared between the two groups. It was found that the total effective rate in group B was higher (92.31% vs. 84.62%) (*P* *<* 0.05). After treatment, the disc height (DH) in group A was obviously lower, and the vertebral body slippage was obviously higher (*P* *<* 0.05) than before. After treatment, there were more patients with nerve root location changes, edema, or disappearance in group B (*P* *<* 0.05). In contrast with JOA and VAS scores before treatment, both the groups showed obvious differences after treatment, especially group B (*P* *<* 0.05). Therefore, the CT images based on the AI algorithm can be used to analyze the treatment effect of LDH, and the scalpel treatment was more effective.

## 1. Introduction

Lumbar disc herniation (LDH) is a common spinal disease [1]. It is usually due to degeneration of the lumbar intervertebral disc, especially the nucleus pulposus. When an external force acts on the lumbar disc, the fibrous ring around the intervertebral disc ruptures easily, and the nucleus pulposus tissue protrudes or prolapses. As a result, the spinal nerve roots are stimulated. Eventually, the patient suffers from local back pain, numbness, and other symptoms [2, 3]. The incidence of LDH is very high and is closely related to factors such as age and occupation. Relevant data show that people aged 25–60 have the highest probability of LDH. In addition, people who have been engaged in labor activities for a long time or have a heavy workload are more likely to have LDH. LDH shows a long course of disease and poor prognosis, and patients are prone to anxiety or emotional disorders, which has a great impact on their quality of life and physical and mental health [4]. The scalpel treatment combines Chinese and Western medicine treatment concepts, showing excellent treatment effect in LDH. In the surgical treatment, a combination of knife and acupuncture is applied to restore the dynamic balance of the lumbar spine, which is extensively adopted in the treatment of lumbar disc herniation [5, 6]. CT imaging is an effective way to diagnose LDH in the clinic [6]. CT images can clearly observe the location and severity of the protrusion of the nucleus pulposus, which is helpful for the doctor's diagnosis and follow-up treatment [7]. Recently, artificial intelligence (AI) in the medical field has become a research hotspot. Modern medical AI based on big data analyzes the examination results through AI methods, which greatly improves the accuracy and sensitivity of diagnosis [8]. The accurate segmentation of medical images is the focus of computer artificial vision. Image segmentation is very important for disease diagnosis, three-dimensional visualization, and follow-up treatment. The realization of accurate segmentation helps doctors understand the actual condition of the patient and formulate a reasonable treatment plan [9,10]. Therefore, AI algorithm was adopted in this work to improve and optimize the CT imaging technology. Then, it was applied in the effect analysis of LDH by scalpel treatment. Finally, the changes in CT parameters and clinical efficacy were discussed.

## 2. Materials and Methods

### 2.1. Research Subjects and Grouping

A total of 78 patients with LDH, who were admitted to the hospital from December 2018 to June 2020, were selected as research subjects, including 42 males and 36 females. They were 35–70 years old. All patients were divided into a lateral crypt block treatment group (group A) and a scalpel treatment group (group B) randomly. This experiment had been approved by the ethics committee of the hospital, and the patients signed consent forms.

Inclusion criteria: the patients who met the criteria for diagnosis and efficacy of TCM diseases, patients aged 18–70 years old, patients who underwent CT examination, and patients with complete clinical data.

Exclusion criteria: patients who were determined as non-LDH after imaging diagnosis; patients with mental illness; patients suffering from diabetes, cardiovascular diseases, and tumor diseases; patients with lumbar vertebra compression fracture and lumbar spondylolisthesis; and patients with lumbar spinal stenosis and hypertrophy of ligamentum flavum.

### 2.2. Treatment Methods

Patients in group A were treated with lateral crypt block. Patients in group B were in the prone position, and a soft pillow was placed under the abdomen to expose the waist and position the spinous process according to the bony landmarks. Combined with imaging examination, marking was performed 2 cm to it. Then, the patient's skin was disinfected, and 0.75% lidocaine was used for infiltration. Subsequently, a small needle knife was used to pierce the marked part vertically to the subcutaneous tissue. Then, a vertical dredging and peeling was performed. When the hand of the patient became loose and the ipsilateral lower limb had radiating acid bilge, the needle was withdrawn. The operation was performed at 4–5 locations each time. Patients in groups A and B were treated once a week, with a maximum of five times.

### 2.3. CT Examination

All patients accepted CT examination for lumbar cross-sectional, lateral, and frontal phases before and after treatment. In reexamination, patients were checked with the same inclination angle, spacing, and thickness as the first time, and the changes were analyzed in terms of protrusion size, DH, vertebral body slippage, and nerve root. The method of measuring the size of the protrusion: the patient's CT image was input into the AutoCAD software to measure the area of the protrusion and the spinal canal and calculate the ratio. DH: the patient's CT image was input into eFilm software to detect the distance from the midpoint of the lower edge of the upper vertebral body to the midpoint of the upper edge of the lower vertebral body. Vertebral body slippage: if the vertebral body did not slip, the slippage of the vertebral body was recorded as 0 mm. If the vertebral body slipped, at first, a bisector was made along the lower edge line of the upper vertebral body and the upper edge line of the lower vertebral body so that it was parallel to both. Then, a central axis was made that intersected this bisector at two points. The distance between the two points was vertebral body slippage, which was measured using eFilm software. Finally, the nerve root changes can be obtained according to CT results.

### 2.4. CT Image Segmentation Using AI Algorithm

Firstly, according to the gray distribution characteristics of the vertebral CT image, the gray adjustment function based on the fusion of neighborhood features was used to enhance the image contrast. In addition, the local binary fitting (LBF) algorithm and PreWork algorithm were introduced in this work to process images. The algorithm adjustment function was defined as follows:

(1) $$\begin{array}{c} f_{0}^{\prime }=f_{0}e^{\alpha -0.45}. \end{array}$$

In the above equation, *f*_0_ refers to the gray value of any pixel point, *f*_0_′ is the neighborhood pixel value of this point, *f*_0_′ is an adjustment function, and *α* is a constant and *α*=∑_*i*=0_^8^*f*_*i*_/255*·*9.

After several iterations, the noise of the CT image was reduced and the image quality was improved.

Then, the prediction segmentation of the bone region was performed as shown in Figure 1. First, initialization was performed to get the first frame gray image SI. SI=*I*_mod_^*i*+1^, where *I* was the original image. Then, the active contour algorithm was applied for segmentation. After binarization, *I*_*b*_′ was obtained. After that, the suture area and key points were obtained, and the *i* frame and the *i+1* frame were fused as follows:

(2) $$\begin{array}{c} I_{\mathrm{mod}}^{i+1}=\alpha \cdot I_{b}^{i}+\beta \cdot I_{enh}^{i+1}. \end{array}$$

Then, noise reduction was performed in the suture area.

(3) $$\begin{array}{c} I_{\mathrm{mod}}^{i+1}\left(x,y\right)=\left\{\begin{array}{c} \mu_{1}\cdot I_{\mathrm{mod}}^{i+1}\left(x,y\right),\left(x,y\right)\in Q_{1}\wedge I_{ori}^{i+1}\left(x,y\right)<th,\\ \mu_{2}\cdot I_{\mathrm{mod}}^{i+1}\left(x,y\right),\left(x,y\right)\in Q_{2}\wedge I_{ori}^{i+1}\left(x,y\right)<th. \end{array}\right. \end{array}$$

The value of *i* was updated continuously until *i* = *n*, and the active contour segmentation algorithm was applied to the segment *I*_update(*n*)_′.

The active contour segmentation algorithm was extensively used in medical image segmentation. Among them, the most representative model was the C-V model, which is expressed as follows:

(4) $$\begin{array}{c} A\left(c_{1},c_{2},C\right)=\mu \cdot \text{Length}\left(C\right)+v\cdot Area\left(inside\left(C\right)\right)\\ +\lambda_{1}\int_{\text{inside}\left(C\right)}{\left|\mu_{0}\left(x,y\right)-c_{1}\right|}^{2}\text{d}x\text{d}y+\lambda_{2}\int_{\text{outside}\left(C\right)}{\left|\mu_{0}\left(x,y\right)-c_{2}\right|}^{2}\text{d}x\text{d}y. \end{array}$$

In equation (4), *C* represents a closed curve; *c*_*1*_ and *c*_*2*_ are the average gray values; *λ*_1_, *λ*_2_, *v*, and *μ* are related parameters; Length(*C*) represents the perimeter C; *Area*(*inside*(*C*)) is the coverage of the area; and *μ*_0_(*x*, *y*) represents the corresponding pixel value.

After the curve C was replaced by zero level set *ϕ*(*x*, *y*)=0, the above equation can be expressed as follows:

(5) $$\begin{array}{c} A\left(c_{1},c_{2},\phi \right)=\mu \int_{\Omega }\delta \left(\phi \left(x,y\right)\right)\left|\nabla \phi \left(x,y\right)\right|\text{d}x\text{d}y+v\int_{\Omega }H\left(\phi x,y\right)\text{d}x\text{d}y\\ +\lambda_{1}\int_{\Omega }{\left|\mu_{0}\left(x,y\right)-c_{1}\right|}^{2}H\left(\phi \left(x,y\right)\right)\text{d}x\text{d}y+\lambda_{2}\int_{\Omega }{\left|\mu_{0}\left(x,y\right)-c_{2}\right|}^{2}\left(1-H\left(\phi \left(x,y\right)\right)\right)\text{d}x\text{d}y, \end{array}$$

in which

(6) $$\begin{array}{c} H\left(\phi \left(x,y\right)\right)=\left\{\begin{array}{c} 1,\phi \left(x,y\right)\geq 0,\\ 0,\phi \left(x,y\right)<0, \end{array}\right.\\ \delta \left(\phi \left(x,y\right)\right)=\frac{\text{d}H\left(\phi \left(x,y\right)\right)}{\text{d}\phi \left(x,y\right)}. \end{array}$$

In the above equations, Ω represents the whole image region and H refers to the Heaviside function.

Then, on the basis of C-V model, LBF model was adopted to improve the operation efficiency. The energy function was defined as follows:

(7) $$\begin{array}{c} E_{x}^{\text{LBF}}\left(C,g_{1}\left(x\right),g_{2}\left(x\right)\right)=\lambda_{1}\int_{\text{in}\left(C\right)}K\left(x-y\right){\left|I\left(y\right)-g_{1}\left(x\right)\right|}^{2}\text{d}y+\lambda_{2}\int_{\text{out}\left(C\right)}K\left(x-y\right){\left|I\left(y\right)-g_{2}\left(x\right)\right|}^{2}\text{d}y. \end{array}$$

In equation (6),K is the kernel function, C stands for contour of image domain Ω, *g*_1_(*x*) and *g*_2_(*x*) are the average fitting values of pixel grays, and *x* is the center point.

The global energy function was expressed as follows:

(8) $$\begin{array}{c} E\left(C,g_{1},g_{2}\right)=\int_{\Omega }E_{x}^{\text{LBF}}\left(C,g_{1}\left(x\right),g_{2}\left(x\right)\right)\text{d}x. \end{array}$$

### 2.5. Observation Indexes

The LDH evaluation form was divided into four levels: cured, markedly effective, effective, and ineffective. 80%–100% improvement rate indicated “cured,” 60%–80% indicated “markedly effective,” 5%–60% indicated “effective,” and less than 25% indicated “invalid”.

Visual analogue scale (VAS) was applied to evaluate the patient's pain before and after treatment, and JOA was to evaluate the improvement of patients' lumbar function.

### 2.6. Statistics

The data were processed by SPSS20.0. *t*-test and independent *t*-test were for intragroup comparison and comparison between groups, respectively. *χ*^2^ test was applied to compare data between groups. The mean ± standard deviation (x(−) ±*s*) illustrated how to calculate measurement data. If *P* *<* 0.05, the difference was statistically significant.

## 3. Results

### 3.1. CT Image Segmentation Results Based on AI Algorithm

Different segmentation algorithms were used to segment the CT images of the lumbar spine (Figure 2). It was evident that the LBF algorithm shrank faster and can segment the vertebral region very well, but the antinoise ability was weak, with poor segmentation effect of regions with strong gray unevenness. Although the PreWork algorithm had perfect antinoise performance and can identify the main bone area, it was not ideal for processing weak edges. In contrast with the above two algorithms, the AI algorithm proposed in this work had the best CT image segmentation effect.

### 3.2. Clinical Data of LDH Patients

Comparison of clinical data was shown in Table 1. There were 22 males and 17 females in group A, aged 35–70 years old, with the average age of 54.34 ± 12.39 years. The course of the disease was within 16–12 years, and the average course of the disease was 2.7 ± 4.8 (months). The VAS score was 5.13 ± 0.76 (points). Group B included 20 males and 19 females, who were 37–68 years old, with an average age of 53.53 ± 10.26 (years). The course of disease was within 14 days–10 years, the average course of disease was 2.5 ± 4.5 (months), and the VAS score was 5.14 ± 0.74 (points). It was evident that there was no notable difference in terms of gender, age, course of disease, and VAS score between the two groups (*P* *>* 0.05).

### 3.3. Comparison of Clinical Efficacy

Figures 3 and 4 presented the clinical efficacy of the two groups. As shown in Figure 3, in group A, there were 7 cured patients, 10 markedly effective patients, 16 effective patients, and 6 ineffective patients. In group B, there were 9 cured patients, 17 markedly effective patients, 10 effective patients, and 3 ineffective patients. It was evident from Figure 4 that the total effective rate of group B was higher (92.31% vs. 84.62%) (*P* *<* 0.05).

### 3.4. Comparison of Quantitative Changes in CT Characteristics

The comparison of the protrusion size before and after treatment was shown in Figure 5. It was evident that the protrusion size of group A before treatment was 0.299 ± 0.123 (cm^2^) and that after treatment was 0.297 ± 0.131 (cm^2^); in group B, that before and after treatment was 0.300 ± 0.119 (cm^2^) and 0.298 ± 0.128 (cm^2^), respectively. There was no notable difference in the size of the protrusions before and after treatment (*P* *>* 0.05).

Figure 6 presented the comparison of DH before and after treatment between the two groups. The DH of group A after treatment was lower (12.98 ± 2.21 (mm) vs. 12.20 ± 2.06 (mm)) (*P* *<* 0.05), while there was no notable difference in the DH of group B before and after treatment (12.87 ± 2.14 (mm) vs. 12.53 ± 2.34 (mm)) (*P* *>* 0.05).

The comparison results of vertebral body slippage before and after treatment are shown in Figure 7. The vertebral body slippage in group A was higher after treatment (1.14 ± 0.51 (%) vs. 0.47 ± 0.33 (%)) (*P* *<* 0.05). In group B, there was notable difference in vertebral body slippage before and after treatment (0.48 ± 0.35 (%) vs. 0.53 ± 0.36 (%)) (*P* *>* 0.05).

### 3.5. Comparison of CT Nerve Root Characteristics

Figure 8 showed the comparison of nerve root positions between the two groups after treatment. 2 cases in group A had changed nerve root position and 37 cases had no change; in group B, 8 cases had changed position and 31 cases had no change. The number of patients with changed nerve root position after treatment in group B was obviously higher (*P* *<* 0.05).

Figure 9 showed the comparison of nerve root edema after treatment between the two groups. There were 18 patients with nerve root edema or disappearance in group A and 10 cases without change; in group B, there were 25 patients with nerve root edema or disappearance and 7 cases without change. The number of patients with nerve root edema or disappearance after treatment in group B was obviously higher (*P* *<* 0.05).

### 3.6. Comparison of VAS Score and JOA Score

Figure 10 showed the VAS score before and after treatment. The VAS score before treatment in group A was 5.13 ± 0.76 (points) and that after treatment was 2.92 ± 0.86 (points); the VAS score before and after treatment in group B was 5.14 ± 0.74 (points) and 2.34 ± 0.89 (points), respectively. The VAS scores of both the groups after treatment were lower than before (*P* *<* 0.05). For comparison between groups, the VAS score of group B after treatment was obviously lower (*P* *<* 0.05).

Figure 11 was the JOA score before and after treatment. The JOA score before treatment in group A was 18.65 ± 1.42 (points) and after treatment was 20.82 ± 1.65 (points); in group B, the JOA score before and after treatment was 18.43 ± 1.67 (points) and 21.89 ± 1.69 (points), respectively. The JOA scores of both groups increased after treatment (*P* *<* 0.05). For comparison between groups, the JOA score of group B after treatment was obviously higher (*P* *<* 0.05).

## 4. Discussion

Traditional clinical diagnosis and treatment are mainly based on the doctor's own experience, with auxiliary examinations. In modern medical technologies, AI technology has been widely used in medical imaging diagnosis, which can assist doctors to obtain the best treatment method. In the study, AI algorithm was adopted to improve and optimize the medical image segmentation. It was found that compared to the LBF algorithm and the PreWork algorithm, the AI algorithm had better results for CT image segmentation. This was consistent with the research results of Minnema et al. (2018) [11], indicating that the segmentation method based on AI algorithm can improve the accuracy of medical CT image segmentation. LDH is a clinically common degenerative spine disease, which will adversely affect the quality of life and work ability of patients. Lateral crypt block treatment can converge drugs at the site of the lesion, thereby effectively eliminating nerve root inflammation and edema, which is an effective nonsurgical treatment [12]. The scalpel treatment can release the patient's bone fibrous tube, supraspinous and interspinous ligaments, facet joint capsule, etc.; reduce the pressure in the facet joint capsule and bone fibrous tube; and relieve joint capsule swelling. At the same time, the treatment method also enlarges the intervertebral foramen, thereby improving ligament ischemia, hypoxia, contracture, and adhesion and promoting the balance of traction between the vertebral ligaments so that the spine is in a balanced state [13]. A large number of studies have shown that scalpel treatment is effective and safe in the treatment of LDH [14, 15]. In the study, it was observed that the total effective rate of group B patients was obviously higher (92.31% vs. 84.62%) (*P* *<* 0.05). For intragroup comparison, after treatment, the DH of group A was obviously lower, and the vertebral body slippage was obviously higher (*P* *<* 0.05). For comparison between groups, in group B, after treatment, the number of patients with nerve root position changes, and nerve root edema or disappearance was obviously higher (*P* *<* 0.05). This revealed that the clinical efficacy of scalpel treatment was better than that of lateral crypt block. This was consistent with the research results of Qiu et al. [16]. Because lateral recess nerve block can only exert anti-inflammatory and analgesic effects, while scalpel treatment not only helps to adjust the mechanical balance of the lumbar spine but also effectively blocks spinal instability, the patient's intervertebral foramina is fully released. Further, this method can also greatly increase the range of nerve root activity. As a result, the nerve root shifts to avoid protrusions, and ultimately, the treatment of LDH is realized. In this study, VAS and JOA scales were used to evaluate the pain improvement and the lumbar function recovery effect. It was found that after treatment, the VAS scores of both the groups decreased (*P* *<* 0.05), with group B having a lower score (*P* *<* 0.05). After treatment, JOA scores of both the groups increased than before (*P* *<* 0.05), with group B having a higher score (*P* *<* 0.05). This indicated that both lateral crypt nerve block and scalpel treatment can effectively treat LDH patients, relieve pain, and improve lumbar function, but scalpel treatment is more effective. This was consistent with the research results of Tang et al. [17].

## 5. Conclusion

In this study, the AI algorithm was used to optimize CT images and analyze the therapeutic effect of scalpel treatment of LDH. It was found that compared with traditional segmentation algorithms, the AI algorithm had the best segmentation effect. What is more, the clinical effect of scalpel treatment was more effective than lateral crypt block treatment. However, there are still some shortcomings in this study. For example, the patient's pain tolerance results are subjective, and the number of samples is limited. In the future, the number of samples should be increased and grouping studies should be conducted on patients with different courses of disease to further analyze the diagnosis of LDH. In short, the results of this study can provide a reference for the imaging diagnosis of LDH.

## Figures and Tables

**Figure 1:** The prediction segmentation flowchart of skeleton area.

**Figure 2:** Comparison on CT image segmentation effects of different algorithms. (a) LBF algorithm; (b) PreWork algorithm; (c) AI algorithm.

**Figure 3:** Comparison of clinical efficacy. 1–4 shows the number of cured, markedly effective, effective, and ineffective patients, respectively.

**Figure 4:** Comparison of total effective rate.  ^*∗*^indicates obvious differences in contrast with group A *P* *<* 0.05.

**Figure 5:** Comparison of protrusion size before and after treatment.

**Figure 6:** Comparison of DH before and after treatment.  ^*∗*^indicates notable differences in contrast with before treatment, *P* *<* 0.05.

**Figure 7:** Comparison of vertebral body slippage before and after treatment.  ^*∗*^indicates notable differences in contrast with before treatment, *P* *<* 0.05.

**Figure 8:** Comparison of nerve root position changes after treatment. # means the difference was statistically obvious in contrast to group A *P* < 0.05.

**Figure 9:** Comparison of cases with nerve root edema after treatment, # means the difference was statistically obvious in contrast to group A *P* < 0.05.

**Figure 10:** VAS score comparison.  ^*∗*^indicates notable differences in contrast with before treatment, *P* *<* 0.05; # indicates notable differences in contrast with group A *P* *<* 0.05.

**Figure 11:** JOA score comparison.  ^*∗*^indicates notable differences in contrast with before treatment, *P* *<* 0.05; # indicates notable differences in contrast with group A *P* *<* 0.05.

**Table 1:** Comparison of clinical data of patients with LDH.

	Group A (*n* = 39)	Group B (*n* = 39)	*P*
Gender (male/female)	22/17	20/19	0.073
Age (years)	35–70	37–68	—
Average age (years)	54.34 ± 12.39	53.53 ± 10.26	0.117
Course of disease	16d − 12 years	14d–10 ears	—
Average course of disease (months)	2.7 ± 4.8	2.5 ± 4.5	0.126
VAS score (point)	5.13 ± 0.76	5.14 ± 0.74	0.035

## Data Availability

The data used to support the findings of this study are available from the corresponding author upon request.
